The article "Comprehensive Analysis of circRNA-Mediated ceRNA Regulatory Networks in relation to Recurrent Implantation Failure" was retracted in 2023. Reasons: unreliable results or conclusions; concerns about the data; concerns about the peer review; concerns about the citations.

# Comprehensive Analysis of circRNA-Mediated ceRNA Regulatory Networks in relation to Recurrent Implantation Failure

**DOI:** 10.1155/2022/8314838

**Published:** 2022-08-23

**Authors:** Hanbing Wang, Wei Lv, Yilin Zhu

**Affiliations:** Department of Gynecology and Obstetrics, Wuhan No. 1 Hospital, Wuhan, China

## Abstract

Recurrent implantation failure (RIF) is attributed to endometrial receptivity dysfunction with many unanswered questions. Up to now, there is no explanation for RIF, and therapeutic strategies are usually limited to supportive care. In this study, we differentially analyzed the raw data deposited in three eligible microarray datasets, GSE111974, GSE121219, and GSE147442 to screen DE-mRNAs, DE-miRNAs, and DE-circRNAs, respectively. The value of log2-fold change |log2FC| ≥ 1 and the adjusted *p* value < 0.05 were considered differentially expressed between RIF and fertile control. We found 350 DE-mRNAs, 43 DE-miRNAs, and 1968 DE-circRNAs between RIF and fertile control. The PPI network identified 6 hub genes with degree ≥10, KDR, AGT, POSTN, TOP2A, RRM2, and PTGS2, in RIF. KDR, AGT, POSTN, TOP2A, and RRM2 were downregulated in endometrial tissue samples of RIF compared with those of fertile control, while PTGS2 was upregulated in endometrial tissue samples of RIF compared with those of fertile control. According to the ceRNA hypothesis, 15 groups of ceRNA network based on 10 circRNAs, hsa_circ_001572, hsa_circ_001884, hsa_circ_001375, hsa_circ_001449, hsa_circ_000029, hsa_circ_001168, hsa_circ_000210, hsa_circ_001484, hsa_circ_001698, and hsa_circ_000089 were constructed in RIF. In conclusion, the present study examined the possible role of circRNAs and their related ceRNA network involved in the pathogenesis of RIF.

## 1. Introduction

Recurrent implantation failure (RIF), as a common condition of embryo implantation failure, has always been a major challenge in assisted reproductive technology. Although RIF is not clearly defined, it is widely accepted that RIF is a failure experience that cannot be successfully implanted in the presence of three or more transfers with high-quality embryos or ten or more transfers of embryo [1, 2]. Embryo factors affecting the pregnancy rate have always been emphasized to be closely related to the cause of RIF [3]. When other parameters such as the number and quality of oocytes and embryos have been used as success parameters, RIF is particularly frustrating for couples. However, the interaction between the embryo and the endometrium, concerning the cell growth and differentiation of the embryo and endometrium, is an important process affecting implantation [4]. Recent evidences indicated that endometrial receptivity dysfunction primarily contributed to the occurrence of RIF [2], and related-biomolecules levels, such as MUC1 [5], HOXA-10, and E-cadherin [6], were found to be altered in women with RIF. However, the underlying mechanism of RIF has not been fully revealed in previous studies, and hence further research is urgently needed to find biomarkers for the diagnosis and prognosis of RIF.

The article "Comprehensive Analysis of circRNA-Mediated ceRNA Regulatory Networks in relation to Recurrent Implantation Failure" was retracted in 2023. Reasons: unreliable results or conclusions; concerns about the data; concerns about the peer review; concerns about the citations.

Extensive studies have demonstrated that messenger RNA (mRNA) encoding protein and noncoding RNA (ncRNA) regulating cell physiology and shape cellular functions such as microRNA(miRNA), long noncoding RNA (lncRNA), and circular RNA (circRNA) were involved in biological processes [7, 8]. CircRNA, as a new class of ncRNA, exhibits high stability, abundance, and tissue specificity. It participates in the process of gene translation into protein and interacts with RNA binding protein through sponging miRNA [9]. Differentially expressed circRNAs were revealed in patients with RIF, indicating the potential of circRNA as biomarkers for clinical diagnosis and treatment of RIF [10]. Construction of competing endogenous RNA (ceRNA) regulatory networks mediated by circRNA to explore candidate genes and circRNA mechanism in various diseases has been established. The hsa_circ_0011385 was confirmed as a ceRNA associated with pathogenesis of bladder cancer via construction of circRNA-miRNA-mRNA regulatory network [11]. As for patients with RIF, hsa_circ_0038383-mediated ceRNA network based on prediction of circRNA–miRNA and miRNA–mRNA pairs was constructed [12]. Nevertheless, the regulatory mechanism of ceRNA network in RIF is still lack of numerous studies.

The present study obtained differently expressed mRNAs, miRNAs, and circRNAs from three databases including GSE111974, GSE121219, and GSE147442 and discussed the prominent circRNAs and their molecular mechanisms in RIF.

## 2. Methods

### 2.1. Retrieval of Microarray Datasets

The GEO database was searched to obtain eligible microarray datasets which must be sourced from human endometrial tissue samples, profiled by same technology, and supplemented with clear series matrix files and gene symbols. Three eligible microarray datasets, GSE111974, GSE121219, and GSE147442, were employed to screen DE-mRNAs, DE-miRNAs, and DE-circRNAs. The GSE111974 dataset, generated on the GPL17077 platform, contains endometrial tissue samples obtained from 24 patients with RIF and 24 fertile control patients. The GSE121219, generated on the GPL18058 platform, includes endometrial tissue samples derived from 8 RIF patients and 10 matched controls. GSE147442, generated on the GPL21825 platform, involves endometrial tissue samples sourced from 8 RIF patients and 8 fertile control patients. The value of log2-fold change |log2FC| ≥ 1 and the adjusted *p* value < 0.05 both were used to evaluate differential expression. The visualization of DE-mRNAs, DE-miRNAs, and DE-circRNAs was presented on the volcano plots and heatmaps.

The article "Comprehensive Analysis of circRNA-Mediated ceRNA Regulatory Networks in relation to Recurrent Implantation Failure" was retracted in 2023. Reasons: unreliable results or conclusions; concerns about the data; concerns about the peer review; concerns about the citations.

### 2.2. Functional Enrichment Analysis

Gene Ontology (GO) and Kyoto Encyclopedia of Genes and Genomes (KEGG) enrichment analyses were carried out for DE-mRNAs in endometrial tissue samples between RIF and fertile control. GO terms are typically classified into the biological process (BP), cellular component (CC), and molecular function (MF), and the KEGG pathway database encompasses biochemical pathways obtaining metabolic and regulatory pathways where the enrichment of DE-mRNAs was determined by *p* value < 0.05 using the “clusterProfiler” software package in the R/Bioconductor.

### 2.3. PPI Network Construction and Hub-Gene Identification

A PPI network was built on the basis of DE-mRNAs in endometrial tissue samples between RIF and fertile control using the STRING tool, whose visualization was accomplished using Cytoscape software (v3.9.0). The high confidence for the interaction score was set as 0.4. The Cytoscape plugin “MCODE” was used to identify significant modules and hub genes, with cut-off criteria of degree ≥10.

### 2.4. Construction of the circRNA-miRNA-mRNA ceRNA Network

1. A computer-based miRNA-mRNA target prediction was performed by mapping hub genes with degree ≥10 in the PPI network into the starBase database.
2. Venn intersection was carried out to screen overlapping miRNAs between targeted miRNAs and DE-miRNAs (GSE121219) in endometrial tissue samples between RIF and fertile control. The intersection follows the principle of miRNA-mRNA regulation, namely, miRNAs posttranscriptional gene silencing by guiding mRNA degradation or translational repression.
3. A computer-based circRNA-miRNA target prediction was also performed by mapping overlapping miRNAs above into the starBase database.
4. Venn intersection was carried out to screen overlapping circRNAs between targeted circRNAs and DE-circRNAs (GSE147442) in endometrial tissue samples between RIF and fertile control. The intersection follows the principle of ceRNA hypothesis that circRNAs share miRNA binding sites and compete for posttranscriptional control of mRNAs.

## 3. Results

### 3.1. Identification of DE-mRNAs between RIF and Fertile Control

The raw data of GSE111974 were differentially analyzed, and mRNAs with a value of log2-fold change |log2FC| ≥ 1 and the adjusted *p* value < 0.05 were considered differentially expressed between RIF and fertile control. We then identified 350 DE-mRNAs consisting of 200 upregulated mRNAs and 150 downregulated mRNAs in endometrial tissue samples of RIF compared with those of fertile control, and all were displayed by the volcano plot (Figure 1(a)) and heatmap (Figure 1(b)).

The article "Comprehensive Analysis of circRNA-Mediated ceRNA Regulatory Networks in relation to Recurrent Implantation Failure" was retracted in 2023. Reasons: unreliable results or conclusions; concerns about the data; concerns about the peer review; concerns about the citations.

### 3.2. GO Annotation and KEGG Pathway Analyses of DE-mRNAs

To evaluate the main functional pathways in RIF, we conducted GO annotation and KEGG pathway analyses of 350 DE-mRNAs between RIF and fertile control. After GO analysis, we found that 350 DE-mRNAs were significantly enriched in 69 GO terms including 60 terms belonging to BP, 3 terms belonging to CC, and 6 terms belonging to MF (Table 1, *p* < 0.05). After KEGG pathway analysis, we found that 350 DE-mRNAs were significantly enriched in 19 KEGG pathways (Table 2, *p* < 0.05).

### 3.3. Identification of Hub Genes

We subsequently construct a PPI network by mapping 350 DE-mRNAs between RIF and fertile control into the STRING database (Figure 2), in which 6 hub genes were identified with degree ≥10, namely, KDR, AGT, POSTN, PTGS2, TOP2A, and RRM2. KDR, AGT, POSTN, TOP2A, and RRM2, were downregulated in endometrial tissue samples of RIF compared with those of fertile control, while PTGS2 was upregulated in endometrial tissue samples of RIF compared with those of fertile control.

### 3.4. Identification of DE-miRNA and Hub Gene Interactions in RIF

We searched the starBase database for putative miRNAs based on KDR, AGT, POSTN, PTGS2, TOP2A, and RRM2. Then, we differentially analyzed the raw data of GSE121219 and identified 43 DE-miRNAs in which there were 22 upregulated miRNAs and 21 downregulated miRNAs in endometrial tissue samples of RIF compared with those of fertile control, and all were displayed by the volcano plot (Figure 3(a)) and heatmap (Figure 3(b)). Three miRNAs (hsa-miR-424-5p, hsa-miR-195-5p, and hsa-miR-29b-3p) targeted KDR and are differentially expressed in RIF. Two miRNAs, hsa-miR-29b-3p and hsa-miR-30c-5p, target POSTN and differentially expressed in RIF. Two miRNAs (hsa-miR-3142 and hsa-miR-30c-5p) targeted RRM2 and are differentially expressed in RIF.

### 3.5. Identification of DE-circRNA and DE-miRNA Interactions in RIF

Subsequently, we differentially analyzed the raw data of GSE147442 and identified 1048 downregulated circRNAs along with 920 upregulated circRNAs in endometrial tissue samples of RIF compared with those of fertile control, all displayed by the volcano plot (Figure 4(a)) and heatmap (Figure 4(b)). Concurrently, we independently mapped hsa-miR-424-5p, hsa-miR-195-5p, hsa-miR-29b-3p, hsa-miR-30c-5p, and hsa-miR-3142 into the starBase database to obtain putative circRNAs. We selected overlapping ones between DE-circRNAs and putative circRNAs that must show the same expression patterns as KDR, POSTN, and RRM2 in RIF by Venn functional intersection. Accordingly, a total of 10 circRNAs, hsa_circ_001572, hsa_circ_001884, hsa_circ_001375, hsa_circ_001449, hsa_circ_000029, hsa_circ_001168, hsa_circ_000210, hsa_circ_001484, hsa_circ_001698, and hsa_circ_000089, stood out.

The article "Comprehensive Analysis of circRNA-Mediated ceRNA Regulatory Networks in relation to Recurrent Implantation Failure" was retracted in 2023. Reasons: unreliable results or conclusions; concerns about the data; concerns about the peer review; concerns about the citations.

### 3.6. Final Construction of the ceRNA Network in RIF

Based on the above DE-miRNA and hub gene interactions, DE-circRNA and DE-miRNA interactions, we constructed 15 groups of the ceRNA network which were involved in RIF (Figure 5).

## 4. Discussion

In recent years, an increasing number of women choose to delay pregnancy, which reduces the success rate of natural pregnancy, leading to an increase in the demand for assisted reproductive technology. Thanks to the advancement of ovarian stimulation, in vitro fertilization embryo transfer has been extensively used as an effective method to treat infertility from the previous evidence [13,14]. However, RIF still remains a challenging issue in assisted reproductive technology, which makes medical staff and patients frustrated. Therefore, new approaches for RIF are urgently needed.

As reported in previous studies, RIF is closely related to endometrial receptivity and related proteins in the endometrium expressed abnormally in patients with RIF [5,15]. miRNA is a small endogenous RNA and a key regulator of posttranscriptional gene expression and candidate genes acting as biomarkers in diseases [16]. Wang et al. revealed that several miRNAs such as miRNA489, miRNA199 A, and miRNA369-3P were considered as the key regulatory factors during RIF through targeting mRNAs [17]. Furthermore, a study presented by Zhou et al. showed that the abnormal expression level of circRNAs in the endometrium of RIF patients was detected [18]. More and more studies have focused on the function and mechanism of circRNAs by constructing the ceRNA network since ceRNA hypothesis was first proposed [19, 20].

In this study, we constructed a circRNA–miRNA–mRNA regulatory network based on three eligible microarray datasets (GSE111974, GSE121219, and GSE147442). It was found that 350 DE-mRNAs were identified in endometrial tissue of RIF patients and fertile control and were performed by GO and KEGG analyses to evaluate the main functional pathways in RIF. We observed that these DE-mRNAs were significantly enriched in 69 GO terms and 19 KEGG pathways. As for GO terms, DE-mRNAs were mainly the enrichment in “axon development,” “apical part of cell,” “endopeptidase inhibitor activity,” and “endopeptidase regulator activity.” KEGG pathway analysis indicated that the phospholipase D signaling pathway and calcium signaling pathway were the top two pathways for these DE-mRNAs. Although there were few reports on phospholipase D directly related to RIF, Kashir et al. manifested that defects of phospholipase C exhibited negative impacts on RIF patients undergoing fertility treatments [20]. Calcium plays a key role in the reproductive process from germ cell maturation to placental development, and the calcium signaling pathway participates in establishment of embryo implantation and pregnancy [21, 22]. Subsequently, we identified 6 hub genes from the PPI network and interaction between DE-miRNAs and hub genes in RIF. The analysis showed that levels of five genes (KDR, AGT, POSTN, TOP2A, and RRM2) were decreased, while PTGS2 was increased in endometrial tissue of RIF compared with those of fertile control. In addition, three miRNAs (hsa-miR-424-5p, hsa-miR-195-5p, and hsa-miR-29b-3p) targeting mRNA KDR were differentially expressed in RIF. Two miRNAs (hsa-miR-29b-3p and hsa-miR-30c-5p) targeted mRNA POSTN and were differentially expressed in RIF. Two miRNAs (hsa-miR-3142 and hsa-miR-30c-5p) targeted RRM2 and are differentially expressed in RIF. Andraweera et al. [23] revealed that KDR expression was reduced in placentae of females with adverse pregnancy outcomes such as preeclampsia, gestational hypertension, and small for gestational age infants. A study on bovine preimplantation embryonic development pointed out that mRNA POSTN was identified in in vitro culture media as an indicator of embryo quality [24]. RRM2 has been widely explored in cancer diseases, and its expression was found to be increased in women with endometriosis-associated ovarian cancer while reduced in women with endometriosis [25]. Based on the DE-circRNA and DE-miRNA interactions in RIF, there were several circRNAs showing same expression patterns as KDR, POSTN, and RRM2 in RIF were identified, including hsa_circ_001572, hsa_circ_001884, hsa_circ_001375, hsa_circ_001449, hsa_circ_000029, hsa_circ_001168, hsa_circ_000210, hsa_circ_001484, hsa_circ_001698, and hsa_circ_000089. Actually, the circRNAs we found were different from the previous evidence revealing circRNAs (hsa_circ_0058161, hsa_circ_0033392, hsa_circ_0030162, hsa_circ_0004121, hsa_circ_0034642, and hsa_circ_0034762) participate in pathogenesis of RIF [26]. It suggested that our circRNAs might be novel biomarkers of RIF.

The article "Comprehensive Analysis of circRNA-Mediated ceRNA Regulatory Networks in relation to Recurrent Implantation Failure" was retracted in 2023. Reasons: unreliable results or conclusions; concerns about the data; concerns about the peer review; concerns about the citations.

In this study, a novel circRNA-miRNA-mRNA regulator network related to RIF was identified, and 10 circRNAs, including hsa_circ_000029, hsa_circ_001168, hsa_circ_000210, hsa_circ_001484, hsa_circ_001698, and hsa_circ_000089, hub-genes, consisting of POSTN, KDR, and RRM2, were involved in the development of RIF. However, the results were only relied on public dataset analysis with small samples, and further clinical experiments are essential to verify our prediction. Moreover, the regulation of circRNAs on miRNAs and miRNAs on hub genes remains unknown. In summary, this work might contribute to explore the initiation and progression of RIF and develop potential treatments for RIF.

## Figures and Tables

**Figure 1:** Identification of DE-mRNAs between RIF and fertile control by differentially analyzing the GSE111974. (a) The volcano plots of DE-mRNAs; (b) The heatmaps showing expression diversity of DE-mRNAs.

**Figure 2:** Construction of PPI network.

**Figure 3:** Identification of DE-miRNAs between RIF and fertile control by differentially analyzing the GSE121219. (a) The volcano plots of DE-miRNAs; (b) The heatmaps showing expression diversity of DE-miRNAs.

**Figure 4:** Identification of DE-circRNAs between RIF and fertile control by differentially analyzing the GSE147442. (a) The volcano plots of DE-circRNAs; (b) The heatmaps showing expression diversity of DE-circRNAs.

**Figure 5:** Final construction of ceRNA network in RIF.

**Table 1:** GO terms significantly enriched by DE-mRNAs between RIF and fertile control.

Ontology	Id	Description	*p*-value	Count
BP	GO:0015849	Organic acid transport	0.008	16
BP	GO:0046942	Carboxylic acid transport	0.008	15
BP	GO:0061564	Axon development	0.008	20
BP	GO:0015711	Organic anion transport	0.008	17
BP	GO:0042310	Vasoconstriction	0.013	8
BP	GO:0044070	Regulation of anion transport	0.013	8
BP	GO:0051047	Positive regulation of secretion	0.013	15
BP	GO:0031667	Response to nutrient levels	0.014	19
BP	GO:0032890	Regulation of organic acid transport	0.014	7
BP	GO:1990822	Basic amino acid transmembrane transport	0.014	4
CC	GO:0045177	Apical part of cell	0.004	19
CC	GO:0016324	Apical plasma membrane	0.009	16
CC	GO:0098862	Cluster of actin-based cell projections	0.046	9
MF	GO:0004866	Endopeptidase inhibitor activity	0.009	11
MF	GO:0030414	Peptidase inhibitor activity	0.009	11
MF	GO:0004867	Serine-type endopeptidase inhibitor activity	0.009	8
MF	GO:0061135	Endopeptidase regulator activity	0.009	11
MF	GO:0061134	Peptidase regulator activity	0.031	11
MF	GO:0005201	Extracellular matrix structural constituent	0.048	9

**Table 2:** KEGG pathways significantly enriched by DE-mRNAs between RIF and fertile control.

Id	Description	*p*-value	Count
hsa04072	Phospholipase D signaling pathway	0.007	7
hsa04211	Longevity regulating pathway	0.011	5
hsa00230	Purine metabolism	0.012	6
hsa00590	Arachidonic acid metabolism	0.013	4
hsa04270	Vascular smooth muscle contraction	0.015	6
hsa04936	Alcoholic liver disease	0.020	6
hsa04920	Adipocytokine signaling pathway	0.020	4
hsa04064	NF-kappa B signaling pathway	0.020	5
hsa04922	Glucagon signaling pathway	0.022	5
hsa04931	Insulin resistance	0.023	5
hsa04514	Cell adhesion molecules	0.024	6
hsa00910	Nitrogen metabolism	0.026	2
hsa04668	TNF signaling pathway	0.026	5
hsa04020	Calcium signaling pathway	0.027	8
hsa05412	Arrhythmogenic right ventricular cardiomyopathy	0.028	4
hsa04152	AMPK signaling pathway	0.034	5
hsa00565	Ether lipid metabolism	0.037	3
hsa01232	Nucleotide metabolism	0.038	4
hsa05410	Hypertrophic cardiomyopathy	0.046	4

The article "Comprehensive Analysis of circRNA-Mediated ceRNA Regulatory Networks in relation to Recurrent Implantation Failure" was retracted in 2023. Reasons: unreliable results or conclusions; concerns about the data; concerns about the peer review; concerns about the citations.

## Data Availability

The data supporting the findings of this study are included within the article.
